The article "Postoperative Curative Effect of Cardiac Surgery Diagnosed by Compressed Sensing Algorithm-Based E-Health CT Image Information and Effect of Baduanjin Exercise on Cardiac Autonomic Nerve Function of Patients" was retracted in 2023. Reasons: signs of a paper mill; suspected computer-generated content; unreliable results or conclusions; concerns about the data.

# Postoperative Curative Effect of Cardiac Surgery Diagnosed by Compressed Sensing Algorithm-Based E-Health CT Image Information and Effect of Baduanjin Exercise on Cardiac Autonomic Nerve Function of Patients

**DOI:** 10.1155/2022/4670003

**Published:** 2022-01-27

**Authors:** Fei Zeng, Jing Luo, Jin Ye, Hao Huang, Wei Xi

**Affiliations:** ^1^Cardio-Thoracic Surgery, Hospital of Traditional Chinese Medicine Affiliated to Xinjiang Medical University, Urumqi, 830000 Xinjiang, China; ^2^Department of Gastroenterology, Xinjiang Urumqi Hospital of Traditional Chinese Medicine, Urumqi, 830000 Xinjiang, China; ^3^Medical Imaging Department, Hospital of Traditional Chinese Medicine Affiliated to Xinjiang Medical University, Urumqi, 830000 Xinjiang, China

## Abstract

This research was aimed at exploring the effect of CT images reconstructed by optimized compressed sensing algorithm on postoperative diagnosis of patients with hypertensive heart disease and the influence of Baduanjin on cardiac autonomic nerve function. Based on the compressed sensing algorithm, the maximum likelihood expectation maximization algorithm was introduced to optimize it, and the optimization algorithm was established. The optimized algorithm and filtered back projection algorithm (FBP) were compared regarding the root mean squared error (RMSE), peak signal-to-noise ratio (PSNR), and structural similar image metric (SSIM). A total of 126 patients with hypertensive heart disease who underwent CT examination in the hospital were selected as study subjects. According to whether Baduanjin intervention was adopted, patients were divided into observation group (conventional treatment +Baduanjin) and control group (conventional treatment), with 63 patients in each group. The effect of CT examination on postoperative diagnosis was analyzed. Systolic blood pressure (SBP), diastolic blood pressure (DBP), differential pressure (DP), respiratory rate and heart rate (HR), very low-frequency (VLF) power, low-frequency (LF) power, high-frequency (HF) power, total power (TP) of HR variability, and changes in LF/HF of patients before and after treatment were compared. The RMSE of the compressed sensing optimization algorithm (3.28 ± 0.36) was significantly lower than that of the FBP algorithm (9.25 ± 1.03) (*P* < 0.05). The SSIM and PNSR of the compressed sensing optimization algorithm were (0.87 ± 0.10) and (21.22 ± 1.60) dB, respectively. The SSIM was significantly higher than the FBP algorithm (*P* < 0.01), and the PNSR was also higher than the FBP algorithm (*P* < 0.05). The detection rate of CT for pleural effusion was 16 cases (25.40%) higher than 5 cases (7.94%) with TTE (*P* < 0.01). After treatment, SBP, DBP, HR, LF, VLF, LF/HF, and DP values in the observation group were lower than those in the control group (*P* < 0.05), and TP and HF were higher than those in the control group (*P* < 0.05). It suggested that a novel algorithm was established based on compressed sensing algorithm to improve image quality. CT image had important guiding significance for postoperative diagnosis of heart. Baduanjin intervention could improve the integrated function of patient's autonomic nervous system and the regulation ability of the vagus nerve.

## 1. Introduction

E-health CT plays an important role in medical diagnosis. The current e-health CT imaging process requires intensive processing of the scanned information. Due to the large amount of collected data, the postreconstruction takes longer, and the reconstruction speed is obviously slower than the scanning speed, which will cause difficulty in imaging of moving organs or poor imaging quality [1]. At present, many scholars have applied its learning algorithm to the e-health CT image reconstruction process, which has improved the image resolution and reconstruction speed [2]. Compressed sensing (CS) adopts the sparsity of the signal for random sampling and adopts nonlinear methods to reconstruct the e-health image. At present, a large number of studies have applied CT to the diagnosis of patients with hypertension and heart disease. The diagnostic accuracy of CT for heart disease is as high as about 95%, and it can also make dynamic observations of the heart, which can clearly and objectively display the pathological anatomy of congenital heart disease [3]. For postoperative heart disease, CT imaging can observe the patency of the anastomosis after the operation, the position and patency of the artificial blood vessel, and the condition of the peripheral pulmonary artery after the transvalvular patch [4]. However, it is limited by image quality, and the accuracy of postoperative diagnosis needs to be further improved.

Hypertensive heart disease is formed due to poor control of hypertension in patients, which causes abnormal changes in the structure and function of the heart. At present, many studies have applied e-health CT in the diagnosis of patients with hypertensive heart disease. However, there are few studies applying it to postoperative follow-up. Hypertensive heart disease is generally treated with drugs such as angiotensin II receptor antagonists and calcium antagonists, but these drugs have side effects, thus causing poor patient compliance [5]. With the continuous improvement of people's awareness of drug safety, nondrug exercise therapy has been favored by the public in recent years. The Baduanjin exercise combines movement and static, gentle and slow, and loose and tight. It has the effects of coordinating the internal organs, promoting “qi” and blood circulation, and softening the muscles and bones. Many studies have shown that aerobic operation has a significant effect on hypertensive heart disease [6]. Autonomic dysfunction is a secondary change of hypertensive heart disease. It is often manifested as decreased vagus activity and increased sympathetic nerve activity, which in turn triggers the occurrence of cardiovascular events [7]. Aerobic exercise can reduce the excitability of the sympathetic nerve and increase the vagus nerve [8]. As a kind of aerobic exercise, there is few researches on Baduanjin's influence on cardiac autonomic nerve function.

To sum up, at present, there is still a problem of sparsity in compressed sensing algorithm reconstructed images, and there are few studies on the adoption of e-Health CT technology in postoperative diagnosis of hypertensive heart disease and the influence of Baduanjin on cardiac autonomic nerve function. 126 patients with hypertensive heart disease who underwent e-health CT examination were selected as study subjects. Compressed sensing algorithm was optimized and applied to the preoperative and postoperative diagnosis of hypertensive heart disease patients. The patients were further treated with Baduanjin adjuvant therapy, to explore the effect of e-health CT image reconstructed by CS optimization algorithm on postoperative diagnosis of hypertensive heart disease patients and the effect of Baduanjin on cardiac autonomic nerve function. This provided a reference basis for postoperative diagnosis and treatment of heart disease patients.

## 2. Materials and Methods

### 2.1. Research Subjects and Grouping

In this study, 126 patients with hypertensive heart disease who underwent CT examination in hospital from June 2018 to December 2020 were selected as study subjects, and the age range was 18-68 years. All patients underwent preoperative echocardiography while undergoing CT examination and were treated with radical or staged surgery. The patients were divided into observation group and control group according to whether Baduanjin intervention method was adopted, with 63 cases in each group. The control group took conventional heart disease drugs for treatment, and the observation group received a 24-week Baduanjin intervention while taking conventional heart disease drugs. The inclusion criteria: (i) those who were diagnosed with hypertensive heart disease; (ii) those who were between 18 and 70 years old; (iii) those who had previously irregular exercise habits. The exclusion criteria: (i) patients with limb dysfunction; (ii) patients with history of brain injury; (iii) patients with severe diseases such as diabetes and inflammatory diseases; (iv) patients with severe cardiopulmonary liver or kidney dysfunction. The study had been approved by the ethics committee of hospital, and all subjects included in the study had signed an informed consent form.

### 2.2. Process of Compressed Sensing Algorithm

The CT image processing is optimized based on compressed sensing algorithm (as shown in Figure 1). First, expectation maximization algorithm (MLEM) is adopted to iterate the initialized CT image to get the initialized total variation minimization (TVM) image. The increment factor and the gradient and direction of the total variation are calculated. The image is corrected in the negative direction of the gradient, and the final *ε* value is taken to determine the termination of the calculation process or the continued iteration.

### 2.3. CS Optimization Algorithm

The signals collected by most e-health systems are generally not directly sparse, and the signals need to be sparse through transform bases [9]. For a signal of length *L*, the signal is *x*; it is expressed as a linear combination as follows.

(1) $$\begin{array}{c} x=\overset{L}{\underset{i=1}{\sum }}\psi_{1}S_{1}=\psi S,x={\left[x_{1},x_{2},\cdots x_{L}\right]}^{T},\;x\in R^{L}. \end{array}$$

*S* is the sparse coefficient. *ψ* is the sparse basis of *N* × *N*; it is expressed as follows: *ψ* = [*ψ*_1_, *ψ*_2_, ⋯, *ψ*_*L*_].

It is assumed that *X* is a discrete signal with length *L*; if *X* itself is sparse, the observation vector *Y* can be expressed as *Y* = *φX*, where *ψ* is the dimensional observation matrix *M* × *L*. If *X* itself is not sparse, the observation vector *Y* can be expressed as follows.

(2) $$\begin{array}{c} Y=\varphi \psi S=\Theta S. \end{array}$$

Θ is a compressed sensing operator of *M* × *L* that satisfies the condition 1‐*ε* ≤ (‖Θ*ϖ*‖_2_/‖*ϖ*‖_2_) ≤ 1 + *ε*, where *ε* is a constant and *ϖ* is a nonzero vector.

Compressed sensing is a problem of solving underdetermined equations under the condition of satisfying the measured value. It can be solved by the method of minimizing the *A*_0_ norm, which can be expressed as Equation (3), where ‖*S*‖_1_ = ∑_*i*=1_^*n*^*S*_*i*_.

(3) $$\begin{array}{c} \underset{S}{\min}{\left\|S\right\|}_{1}\text{s}.\text{t}.\;y=\varphi \psi S. \end{array}$$

It is assumed that *X* is one-dimensional discrete data with length *L*, which is expressed as an orthogonal basis as follows.

(4) $$\begin{array}{c} B={\left[b_{1},b_{2},\cdots b_{L}\right]}^{T},\;L\in R^{L}. \end{array}$$

It is expressed in the form of a linear combination as follows.

(5) $$\begin{array}{c} X=\overset{L}{\underset{i=1}{\sum }}\psi_{i}S_{i}=\psi S. \end{array}$$

The sparse signal of length *M* obtained after sparse transformation in Equation (5) is expressed as follows.

(6) $$\begin{array}{c} y=\phi x=\phi \psi S=\Theta S,\;\Theta =\phi \psi . \end{array}$$

*ϕ* is the observation matrix *M* × *L*, and *ψ* is the sparse basis.

The finite difference transform is used as the optimization objective function to optimize the CT image, and the two-dimensional total variation function is expressed as follows.

(7) $$\begin{array}{c} T\left(F\right)=\int_{\Omega }\sqrt{{\left|\nabla F\right|}^{2}}dxdy=\int_{\Omega }\sqrt{{\left|\partial F/\partial x\right|}^{2}+{\left|\partial F/\partial y\right|}^{2}}dxdy. \end{array}$$

Based on this function, to obtain faster solution speed and higher stability, it is transformed into

(8) $$\begin{array}{c} T\left(F\right)=\int_{\Omega }\sqrt{{\left|\nabla F\right|}^{2}}dxdy=\int_{\Omega }\sqrt{{\left|\partial F/\partial x\right|}^{2}}dxdy+\int_{\Omega }\sqrt{{\left|\partial F/\partial y\right|}^{2}}dxdy. \end{array}$$

The solution of the reconstructed image *F* is as follows.

(9) $$\begin{array}{c} \min T\left(F\right),\text{S}.\text{t}.P=AF,F\geq 0. \end{array}$$

In Equation (9), *P* is the transmission projection image, *A* is the observation matrix, and *F* is the reconstructed image.

For the initial reconstructed image *F*_0_(*k* = 0) = 0, *k* is the total number of iterations. For the initial reconstructed image *F*_0_, the maximum likelihood estimation algorithm is used to iterate the image. The algorithm is as follows.

(10) $$\begin{array}{c} f_{j}^{k+1}=f_{j}^{k}\frac{1}{\sum_{i}\alpha_{i,\text{j}}}\underset{i}{\sum }\alpha_{i,\text{j}}\frac{p_{i}}{\sum_{i}\alpha_{i,\text{j}}f_{j}^{k}}. \end{array}$$

*k* is the total number of iterations, *f*_*j*_^*k*^ is the estimated value after *k* iterations, *p*_*i*_ is the projection value of the *i*th ray, and *α*_*i*,*j*_ represents the probability of the photon emitted from the object pixel *j* being detected by the *i*th unit of the detector. The nonconstrained calculation method is adopted to calculate the initial reconstructed image *F*.

(11) $$\begin{array}{c} F\left(k\right)\left\{\begin{array}{cc} F_{m}\left(k\right), & F_{m}\left(k\right)\geq 0,\\ 0, & F_{m}\left(k\right)<0. \end{array}\right. \end{array}$$

The increment factor of processed image *F*_*T*_^0^(*k*) = *F*_*P*_(*k*) is calculated via the following equation.

(12) $$\begin{array}{c} E\left(k\right)=\left\|X_{M}^{0}\left(k\right)X_{P}\left(k\right)\right\|. \end{array}$$

Equation (13) is adopted to calculate the gradient and direction of the total variation, and Equation (14) is adopted to further correct the image in the negative direction of the gradient, where *λ* is the adjustment factor, $\bar{G}$ is the total variation gradient, and $\tilde{G}$ is the total variation direction.

(13) $$\begin{array}{c} \bar{G}\left(k-1\right)={\left.\frac{\partial {\left\|F\right\|}_{T}}{\partial f_{i,j}}\right|}_{F=F^{n-1}\left(k\right)},\tilde{G}\left(k\right)=\frac{\bar{G}\left(k\right)}{\left|\bar{G}\left(k\right)\right|}, \end{array}$$

(14) $$\begin{array}{c} F_{T}^{m}\left(k\right)=F_{T}^{m-1}\left(k\right)-\lambda E\left(k\right)\tilde{G}\left(k\right),\;n=n+1. \end{array}$$

The above calculation result satisfies the condition ‖*F*_*P*_^*k*^(*k*) < *F*_*P*_^*k*−1^(*k*)‖ < *ε*, where *ε* is an arbitrarily small positive number.

### 2.4. Image Quality Evaluation Indexes

MSE is taken to evaluate the degree of difference between two sets of data [10]. The MSE calculation method of the two-dimensional image is $\text{MSE}=\left(1/m,n\right)\sum_{i=0}^{m-1}\sum_{j=0}^{n-1}{\left\|I\left(i,j\right)-\tilde{I}\left(i,j\right)\right\|}^{2}$, then the RMSE for the two-dimensional image is expressed as Equation (15), where *I*(*i*, *j*) and $\tilde{I}\left(i,j\right)$ are the two images to be compared.

(15) $$\begin{array}{c} \text{RMSE}=\sqrt{\text{MSE}}=\sqrt{\frac{1}{m,n}\overset{m-1}{\underset{i=0}{\sum }}\overset{n-1}{\underset{j=0}{\sum }}{\left\|I\left(i,j\right)-\tilde{I}\left(i,j\right)\right\|}^{2}}. \end{array}$$

PSNR is often used to evaluate the gap between the image to be estimated and the ideal image [11], and its calculation method is as follows.

(16) $$\begin{array}{c} \text{PSNR}\left(f,g\right)=10\log_{10}\left(\frac{L^{2}}{\text{MSE}\left(f,g\right)}\right). \end{array}$$

In Equation (16), *L* is the peak signal, *f* is the ideal image, *g* is the image to be estimated, MSE(*f*, *g*) is the MSE of the image, MSE(*f*, *g*) = (1/*MN*)∑_*i*=1_^*M*^∑_*j*=1_^*N*^(*f*(*i*, *j*) − *g*(*i*, *j*))^2^, and *M* × *N* is the size of the image to be estimated.

SSIM is a mechanism that combines images when evaluating image quality, and the evaluation results are more similar to human senses [12]. SSIM evaluates image quality mainly from three aspects: brightness, structure, and contrast, among which brightness contrast calculation method is as follows.

(17) $$\begin{array}{c} L\left(f,g\right)=\frac{2\mu_{f}\mu_{g}+c_{1}}{\mu_{f}^{2}+\mu_{g}^{2}+c_{1}}. \end{array}$$

The contrast calculation is as follows.

(18) $$\begin{array}{c} C\left(f,g\right)=\frac{2\sigma_{f}\sigma_{g}+c_{2}}{\sigma_{f}^{2}+\sigma_{g}^{2}+c_{2}}. \end{array}$$

The structural contrast calculation is as follows.

(19) $$\begin{array}{c} S\left(f,g\right)=\frac{2\sigma_{fg}+c_{3}}{\sigma_{f}\sigma_{g}+c_{3}}. \end{array}$$

Then, SSIM is expressed as follows.

(20) $$\begin{array}{c} \text{SSIM}\left(f,g\right)={\left(L\left(f,g\right)\right)}^{\alpha }\cdot {\left(C\left(f,g\right)\right)}^{\beta }•{\left(S\left(f,g\right)\right)}^{\gamma }. \end{array}$$

In Equation (20), *μ*_*f*_, *μ*_*g*_, *σ*_*f*_, and *σ*_*g*_ are the mean value and standard deviation of the ideal image *f* and the image to be evaluated *g*, respectively. *σ*_*fg*_ is the covariances of *f* and *g*, *c*_1_ = (*k*_1_*R*)^2^, and *c*_2_ = (*k*_2_*R*)^2^. *R* is the range of image pixel values. *k*_1_ and *k*_2_ are 0.01 and 0.03, respectively, *c*_3_ = *c*_2_/2, and *α* = *β* = *γ* = 1.

### 2.5. Baduanjin Exercise Intervention Program and Its Detection Indexes

The duration of Baduanjin exercise intervention was 24 weeks, and all observation subjects learned the Qigong Baduanjin for the first time after being included in the research. Intervention methods were mainly divided into three parts: warming-up activity, formal activity, and cooling-down activity. Exercise was mainly moderate intensity of new fitness qigong Baduanjin. The first week was mainly about the decomposition of technical movements to make the subjects form the correct dynamic pattern. In the second week, breathing was added to the action for a complete set of exercises. From the third week, the whole set of movements began to be practiced. The movement frequency was 5 times/week, 40 min/time. The warming-up activity mainly included aerobics and some stretching exercises, 10 min/time. The whole set of Baduanjin movements was practiced during the formal activity time, 2-3 times/time. The cooling-down activity was 10 min/time. The whole training process was conducted under the guidance of professional Baduanjin teacher. The HR of the subjects was measured to reflect the intensity of exercise, and the hospital would uniformly distribute the convenient HR detector. The HR of each subject was measured and recorded immediately after each activity. The HR of the subjects was collected and analyzed every week, the exercise intensity was adjusted according to the changes of the HR of the subjects, and special guidance was given.

### 2.6. Observational Indexes

The autonomic nervous function indexes of SBP, DBP, DP, respiratory rate, and HR were recorded. The VLF power, LF power, HF power, TP of HR variability, and changes in LF/HF of patients before and after treatment were also recorded.

### 2.7. Statistical Methods

The test data was processed via SPSS19.0 statistical software, and measurement data was expressed as mean plus or minus standard deviation ($\overset{¯}{x}\pm s$). The comparison of changes in HR and blood pressure between and within groups before and after intervention was performed by *t* test. Counting data was expressed in percentage (%) and processed by *χ*^2^ test. *P* < 0.05 indicated that the difference was statistically significant.

## 3. Results

### 3.1. Analysis of CT Images Reconstructed by Compressed Sensing Algorithm

The CS optimization algorithm was compared with the FBP algorithm. In Figure 2, the FBP reconstructed image was quite different from the original image, and there were obvious artifacts. The reconstructed image of the CS optimization algorithm was basically small in difference from the original image and basically coincided with the original image.

### 3.2. Evaluation of Image Quality Reconstructed by CS Optimization Algorithm

Under the same conditions, the RMSE of the FBP algorithm and the compressed sensing optimization algorithm was 9.25 ± 1.03 and 3.28 ± 0.36, respectively. The RMSE of the compressed sensing optimization algorithm was significantly lower than that of the FBP algorithm (*P* < 0.05). The SSIM and PNSR of the compressed sensing optimization algorithm were 0.87 ± 0.10 and 21.22 ± 1.60 dB, respectively. The SSIM and PNSR of the FBP algorithm are 0.23 ± 0.03 and 14.39 ± 2.35 dB, respectively. The SSIM value of the compressed sensing optimization algorithm was significantly higher than the FBP algorithm (*P* < 0.01), and the PNSR was also significantly higher than the FBP algorithm (*P* < 0.05) (Figure 3).

### 3.3. CT Image Evaluation of Postoperative Heart

49 cases of all study subjects were treated with radical resection. After treatment (arrow in Figure 4(e)), patient's shunt vessel was unblocked, and the LPA became wider than before treatment (Figure 4(a)). 38 cases underwent correction of aortic arch interruption. Before treatment, the descending part of the middle arterial arch was interrupted (Figure 4(b)). After the treatment, both lungs and a little atelectasis were seen (arrow in Figure 4(f)). 27 cases underwent total vena cava-pulmonary connection. After treatment (Figure 4(g)), the diameter of patient's pulmonary aorta was larger than before (Figure 4(c)). 12 cases underwent shunting. After treatment, the RSVC-RPA connection was unobstructed, the lower right lung was atelectasis (arrow in Figure 4(h)), and the pulmonary artery diameter did not change significantly from that before treatment (Figure 4(d)).

### 3.4. CT Image Evaluation of Postoperative Complications

CT and transthoracic echocardiography (TTE) were adopted to detect postoperative complications of patients, and the differences in the detection of complications between the two were analyzed (Figure 5). CT was adopted to detect postoperative complications. The probability was significantly higher than that of the control group (*P* < 0.05). The detection rate of CT for pleural effusion was 16 cases (25.40%), and the detection rate of TTE was 5 cases (7.94%). The detection rate of CT for pleural effusion was significantly higher than that of TTE (*P* < 0.01).

### 3.5. Comparison of Basic Data of Research Subjects

The basic data of the observation group and the control group were statistically analyzed (Table 1). There was no significant difference between the two groups in basic data such as age, gender, BMI, increase, and weight (*P* > 0.05).

### 3.6. Comparison of HR Variability between Two Groups of Patients before and after Treatment

Before treatment, the observation group and the control group had no significant difference in HR variability indexes of TP, VLF, LF, HF, and LF/HF (*P* > 0.05). After treatment, the HR variability indexes of LF, VLF, and LF/HF values of control group were higher than those in the observation group (Figure 6), and there was a significant difference in LF/HF between the two groups (*P* < 0.05). After treatment, TP and HF of the observation group were higher than those of the control group, with significant difference (*P* < 0.05).

### 3.7. Comparison of Autonomic Nerve Indexes between Two Groups of Patients before and after Treatment

There was no significant difference in SBP, DBP, and DP between the observation group and the control group before treatment (Figure 7). After treatment, the SBP, DBP, and DP values of the observation group were lower than those of the control group, and the SBP and DBP values were significantly different from those of the control group (*P* < 0.05). After treatment, BP, DBP, and DP of the two groups were lower than before treatment (*P* < 0.05). There was no significant difference in respiratory rate and HR between the observation group and the control group before treatment (Figure 8). After treatment, the respiratory rate and HR of both groups decreased (*P* < 0.05). After treatment, the HR of the observation group was significantly lower than the control group (*P* < 0.05).

## 4. Discussion

The FBP algorithm is an analytical algorithm with a faster reconstruction speed, and the reconstructed image of dense angle projection is often taken as the standard for evaluating other algorithms [13]. After the compressed sensing algorithm was optimized, the reconstructed image was compared with those treated by FBP, and it was found that there were obvious artifacts between the FBP reconstructed image and the original image. The CS optimization algorithm reconstructed image basically coincided with the original image. Moreover, the RMSE value of the CS optimization algorithm reconstructed image was lower than those of FBP algorithm (*P* < 0.05), and the SSIM and PNSR values were significantly higher than those of FBP (*P* < 0.05). It was revealed that the difference between the CS optimization algorithm reconstructed image and the original image was small, and the image quality was high. CT scans are faster and can clearly show the complex anatomy of the cardiovascular system [14]. CT technology was applied in the postoperative diagnosis of patients with hypertensive heart disease, and it was found that CT scanning technology could clearly show the changes of patient's preoperative and postoperative lesions. Moreover, the probability of postoperative complications detected by CT was significantly higher than that of ultrasound (*P* < 0.05). Iwamoto et al. (2019) [15] adopted CT angiography technology to observe the position of the artificial blood vessel and the general condition of the anastomosis in patients with congenital heart disease after surgery. It was found that the rate of complications detected by CT was higher than that by ultrasound, which was similar to the results of this article.

At present, most interventions on autonomic nerves focus on drug intervention research [16]. Baduanjin was adopted to intervene in patients and observe the changes in physiological index after treatment. The results showed that after treatment, SBP, DBP, HR, and LF/HF in the observation group were lower than those in the control group (*P* < 0.05), while TP and HF were higher than those in the control group (*P* < 0.05). Some researchers took physiological indexes such as SBP, DBP, HR variability, palm conductivity, pulse pressure difference, and HR to reflect patient's autonomic nerve response to harmful stimuli. It was found that the SBP, DBP, pulse pressure difference, and HR under the induced emotion would all decrease [17], which was similar to this research results. It was revealed that Baduanjin intervention could improve the overall integration function of patient's autonomic nervous system and improve the regulation and control ability of the vagus nerve.

## 5. Conclusion

To explore the effect of electronic medical CT images reconstructed by compressed sensing optimization algorithm on postoperative diagnosis of hypertensive heart disease patients and the influence of Baduanjin on cardiac autonomic nervous function, the optimization algorithm was established based on the compressed sensing algorithm and applied to the diagnosis of cardiac postoperative efficacy. The results showed that the compression sensing based optimization could improve CT image quality. Baduanjin intervention could significantly reduce SBP, DBP, HR, and LF/HF, and improve TP and HF levels. The overall integration function of autonomic nervous system and vagal nerve regulation ability were improved. However, there are still some shortcomings in this work. Only FBP algorithm is used in the optimization of compressed sensing algorithm results analysis, and it is not compared with other iterative reconstruction algorithms. In the later research, the optimization algorithm in this work will continue to be compared and analyzed with other algorithms. In conclusion, this study provides a reference for the diagnosis and treatment of cardiac surgery.

## Figures and Tables

**Figure 1:** The basic flow and optimization of the adaptive ultrasound imaging algorithm.

**Figure 2:** Comparison of CT image reconstruction results with different algorithms ((a) the reconstructed result of FBP algorithm and the horizontal center profile of the original image; (b) the reconstructed result of FBP algorithm and the vertical center profile of the original image; (c) the reconstructed result of CS optimization algorithm and the horizontal center profile of the original image; (d) the reconstructed result of CS optimization algorithm and the vertical center profile of the original image).

**Figure 3:** Comparison of reconstructed image quality with different algorithms (^∗^ indicated a significant difference compared with the FBP algorithm, *P* < 0.05; ^∗∗^ indicated a very significant difference compared with the FBP algorithm, *P* < 0.01).

**Figure 4:** Preoperative and postoperative CT image evaluation of the heart ((a) TOF basic lesions of the patient; (b) the unnamed artery branched out from the subclavian artery and the shunt was not smooth before treatment; (c) localized narrowing of the descending part of the arterial arch before treatment; (d) the descending aortic arch was severed before treatment; (e) the shunt vessel was unblocked after treatment; (f) both lungs exuded with a little atelectasis after treatment; (g) the diameter of the pulmonary aorta increased after treatment; (h) right superior vena cava-right pulmonary artery connection was unobstructed after treatment).

**Figure 5:** Comparison of the detection rate of postoperative complications between CT and TTE ((a) pulmonary infection; (b) atelectasis; (c) pleural effusion; (d) pericardial effusion; (e) artificial vascular disease; (f) artificial vascular anastomotic disease; (g) pneumothorax; (h) pneumothorax) (^∗∗^ indicates significant difference compared with TTE, *P* < 0.01).

**Figure 6:** Comparison of frequency domain indexes of HR variability before and after treatment between the two groups ((a) comparison of frequency domain indexes between the two groups of patients before treatment; (b) comparison of frequency domain indexes between the two groups of patients after treatment) (^∗^ represents statistical difference compared with the control group, *P* < 0.05).

**Figure 7:** Differences of SBP, DBP, and DP between the two groups of patients before and after treatment ((a) comparison of SBP, DBP, and DP between two groups of patients before treatment; (b) comparison of SBP, DBP, and DP between two groups of patients after treatment) (^∗^ represents statistical difference compared with the control group, *P* < 0.05).

**Figure 8:** Differences in respiratory rate and HR between the two groups of patients before and after treatment ((a) comparison of respiratory rate and HR between two groups of patients before treatment; (b) comparison of respiratory rate and HR between two groups of patients after treatment) (^∗^ represents statistical difference compared with the control group, *P* < 0.05).

**Table 1:** Comparison of basic data of two groups of patients.

Item	Observation group	Control group	*χ* ^2^	*P*
Age (year)	63.56 ± 1.54	61.82 ± 1.23	0.92	0.132
Gender (male/%)	29 (46.03)	31 (49.21)	0.83	0.258
BMI (kg/m^2^)	22.61 ± 0.82	2342 ± 0.71	0.75	0.234
Weight (kg)	67.27 ± 2.94	65.91 ± 3.39	-2.87	0.216
Height (cm)	168.4 ± 9.9	167.6 ± 10.1	1.93	0.225

## Data Availability

The data used to support the findings of this study are available from the corresponding author upon request.
